This article has been retracted.

# Circular RNA (circ)_0129047 upregulates bone morphogenetic protein receptor type 2 expression to inhibit lung adenocarcinoma progression by sponging microRNA (miR)-1206

**DOI:** 10.1080/21655979.2022.2070580

**Published:** 2022-05-16

**Authors:** Xinxin Xue, Yajun Chen

**Affiliations:** Department of Respiratory and Critical Care Medicine, Wuhan Third Hospital & Tongren Hospital of Wuhan University, Wuhan, Hubei, China

**Keywords:** Circ_0129047, miR-1206, BMPR2, lung adenocarcinoma (LAC), proliferation

## Abstract

Circular RNAs (circRNAs) play significant roles in the tumorigenesis and progression of various cancers, including lung adenocarcinoma (LAC). However, their underlying biological functions in LAC remain unclear. Here, we investigated the tumor suppressor role of the newly identified circRNA, circ_0129047, in LAC tumorigenesis and progression. The expression levels of circ_0129047, microRNA (miR)-1206, and bone morphogenetic protein receptor type 2 (BMPR2) mRNA in LAC cells and tissues were monitored using reverse transcription-quantitative polymerase chain reaction. Dual-luciferase reporter, RNA immunoprecipitation, and RNA pull-down assays were used to confirm the targeting relationships among circ_0129047, miR-1206, and BMPR2 mRNA. Functional experiments for A549 and PC9 cells were performed using cell counting kit-8, bromodeoxyuridine enzyme-linked immunosorbent, caspase-3 activity, cell adhesion, wound healing, and transwell assays. Circ_0129047 expression levels were reduced in LAC cells and tissues. Mechanistically, we discovered that circ_0129047 could sponge miR-1206, and miR-1206 could directly target BMPR2. In addition, circ_0129047 or BMPR2 knockdown facilitated the viability, proliferation, adhesion, migration, and invasion, while inhibiting the apoptosis of LAC cells. Furthermore, the inhibitory effects of circ_0129047 or BMPR2 overexpression on the malignant phenotype of LAC cells could be reversed by the overexpression of miR-1206. In conclusion, circ _0129047 was found to play a tumor suppressive role in LAC progression; it upregulated BMPR2 expression to inhibit LAC progression by sponging miR-1206.

**Abbreviations:** non-small cell lung cancer (NSCLC); small cell lung cancer (SCLC); lung adenocarcinoma (LAC); Circular RNA (circRNA); MicroRNA (miRNA); bone morphogenetic protein (BMP); squamous cell lung cancer (SCC); RNA immunoprecipitation (RIP)

## Highlights

- Circ_0129047 and BMPR2 expression levels are decreased in LAC, while miR-1206 levels are increased.
- Circ_0129047 can sponge miR-1206 and release BMPR2.
- Circ_0129047 or BMPR2 knockdown facilitates the malignant behavior of LAC cells.
- Circ_0129047 or BMPR2 overexpression suppresses the malignant phenotype of LAC cells.
- Upregulation of miR-1206 expression promotes LAC progression.

## Introduction

Lung cancer is a leading cause of cancer-related deaths worldwide, posing the biggest threat to human health as the most malignant tumor [1,2]. The incidence of lung cancer and mortality rates associated with it are the highest at 11.6 and 18.4% respectively, as reported in the 2018 statistics [3]. Lung cancer can be classified into two broad categories: non-small cell lung cancer (NSCLC) and small cell lung cancer (SCLC) [4]. NSCLC can be further classified into four types: squamous cell lung carcinoma, large cell lung carcinoma, lung adenocarcinoma (LAC), and others [5]. Among these, LAC is the most common, accounting for approximately 40% of all primary lung cancer cases [6]. Although considerable efforts are being made for the diagnosis and treatment of LAC, the lack of effective screening methods and presence of metastasis have resulted in unsatisfactory survival rates [7], with the five-year survival rate being less than 15% [8,9]. Consequently, further elucidation of the mechanisms underlying the carcinogenesis and progression of LAC is urgently required.

Circular RNA (circRNAs) are a type of non-coding RNAs with multiple features, including closed loop structure and high conservation and stability [10,11]. In recent years, circRNAs have received extensive attention owing to their multiple gene regulatory functions, including sponging of microRNAs (miRNAs), RNA–protein complex formation, and regulation of transcription, splicing, and protein translation [11,12]. CircRNAs play important roles in the pathogenesis and development of some cancer types [13], and circRNA research can enrich our knowledge on cancer and provide new opportunities for cancer treatment. Several circRNAs, such as hsa_circ_0013958 [5], hsa_circ_0001946 [14], hsa_circ_0000326 [15], hsa_circ_0000792 [16], hsa_circ_0006427 [17], and hsa_circ_0012673 [18], play carcinogenic or cancer-inhibiting roles in LAC by sponging miRNAs. Circ_0129047 is a novel circRNA that has not previously been identified in any cancer type, including LAC. Hence, it may be of vital significance to identify circ_0129047 and study its role and regulatory mechanisms in LAC.

miRNAs are small non-coding RNAs consisting of only 18–25 nucleotides [19]. miRNAs can combine with the 3′-untranslated regions (UTRs) and alter the expression of downstream target genes by inducing mRNA degradation or translational inhibition [20,21]. miRNAs exert their carcinogenic or tumor suppressive effects by suppressing cancer-related downstream target genes, and this regulatory role has been identified in many cancer types [22,23]. Several miRNAs play important roles in LAC. For example, miR-938 [24], miR-186-5p [25], and miR-147b [26] promote carcinogenesis, while miR-485 [27], miR-767-3p [28], and miR-198-5p [29] inhibit carcinogenesis. miR-1206 is located in an unstable region of the human genome, on chromosome 8q24, which is a well-known cancer-related region [30–32]. Plasmacytoma variant translocation 1, a gene located in this region, is a key driver of carcinogenesis and encodes six annotated miRNAs, including miR-1206 [32–34]. However, it is unclear whether miR-1206 is a tumor suppressor or promoter. High expression levels of miR-1206 are found in Burkitt lymphoma cells [30], while little or no expression of miR-1206 is detected in cancerous and non-cancerous gastric tissues and cell lines [31] as well as in primary normal and prostate cancer samples [35]. To date, the expression and function of miR-1206 in LAC have not been studied; therefore, it is necessary to investigate the role of miR-1206 in LAC.

Bone morphogenetic protein receptor type 2 (*BMPR2*) is located on chromosome 2q33.1-q33.2, and it consists of 13 exons. It encodes a member of the bone morphogenetic protein (BMP) transmembrane serine/threonine kinase receptor family [36]. BMPs, as ligands of this receptor, are members of the transforming growth factor-β superfamily of signaling molecules and participate in endochondral bone formation, embryogenesis, and oncogenesis [37–39]. As a vital component of BMP signal transduction, BMPR2 plays an important role in the tumorigenesis and development of cancer by acting as a tumor promoter (upregulation) or tumor suppressor (downregulation) [40,41]. *BMPR2* is considered an oncogene in some tumors, including chondrosarcoma [42], osteosarcoma [43,44], and gastric cancer [45]. Furthermore, *BMPR2* expression levels are downregulated in some cancers, such as colon cancer [46], human prostate cancer [47], neuroblastoma [48], bladder transitional cell carcinoma [49], squamous cell lung cancer, and LAC [50]. Although the downregulation of BMPR2 expression has been reported in LAC, the underlying mechanism remains unclear.

The primary objective of the present study was to explore the clinical significance and mechanism of a novel circRNA, circ_0129047, and interaction axis, circ_0129047/miR-1206/BMPR2, in LAC. Our study hypothesized that circ_0129047 upregulated BMPR2 expression to inhibit LAC progression by sponging miR-1206. We expected to obtain a better understanding of the mechanism of LAC tumorigenesis and progression and offer new insights for the treatment and prognosis of LAC.

## Material and methods

### Clinical tissue samples

Frozen samples of LAC tissues and matched para-cancerous non-tumor tissues were obtained from 37 patients with LAC who underwent surgical resection in our hospital. The clinical features of the patients are described in Table 1. None of the patients received any local or systemic treatment prior to surgery. We obtained consent from all patients or their relatives for participation in the study, and all patients signed informed consent forms before surgery. This study was approved by ethics committee of Wuhan Third Hospital & Tongren Hospital of Wuhan University (approval number: 武三医KY2021-031) and all experimental procedures adhered to the rules of the ethics committee.

**Table 1.** The clinical characteristics of patients with lung adenocarcinoma

Characteristics	Case (37)
Age (years)	
≤ 55	(45.9%)
> 55	20 (54.1%)
Gender	
Female	16 (43.2%)
Male	21 (56.8%)
Tumor stage	
T1 or T2	18 (48.6%)
T3 or T4	19 (51.4%)
Node stage	
N0 or N1	17 (45.9%)
N2 or N3	20 (54.1%)
Metastasis	
0	7 (18.9%)
1a	16 (43.2%)
1b	14 (37.8%)

### Cell lines and cell culture

The normal human bronchial epithelial cell line, Beas-2B (Cat#: BNCC338205), and five LAC cell lines, A549 (Cat#: BNCC100215), Calu-3 (Cat#: BNCC338514), H1975 (Cat#: BNCC340345), H460 (Cat#: BNCC339581), and PC9 (Cat#: BNCC340767), were purchased from BeNa Culture Collection (BNCC, China). Dulbecco’s modified Eagle’s minimal essential medium (Gibco, USA) containing 10% fetal bovine serum (FBS) (Gibco, USA) was used to cultivate Beas-2B, Calu-3, and PC9 cells, whereas the Roswell Park Memorial Institute-1640 medium containing 10% FBS (Gibco, USA) was used to cultivate the other cells. All cells were routinely cultured under the same conditions in an incubator containing 5% CO_2_ at 37°C.

### Cell transfection

The miR-1206 mimic (mimic), circ_0129047 overexpression vector (circ-OE), BMPR2-OE, and corresponding negative controls used in this study were purchased from GenePharma (China). Circ_0129047 small interfering RNA (siRNA) (si-circ), BMPR2 siRNA (si-BMPR2), and negative control siRNA (si-NC) were purchased from RiboBio (Guangzhou, China). The OE (100 nM), mimic (100 nM), and siRNA (50 nM) were individually or in combination transfected into A549 and PC9 cells using the Exfect 2000 Transfection Reagent (Cat#: T202-01; Vazyme, China), according to the manufacturer’s instructions. Then 48 h post-transfection, the transfection efficiency in A549 and PC9 cells was assessed by reverse transcription quantitative polymerase chain reaction (RT-qPCR) analysis. The sequences of vectors are listed in Supplementary Table 1.

### RNA isolation and RT-qPCR

TRNzol Universal reagent (Cat#: DP424; TIANGEN, China) was used to lyse the frozen tissues or cultured cells for total RNA isolation and purification. A cytoplasmic and nuclear RNA purification kit (Cat#: NGB-21000; Norgen Biotek, Canada) was used to isolate the nuclear and cytoplasmic RNA from cultured A549 and PC9 cells. RNA concentration and purity were assessed using a SHIMADU UV spectrophotometer (Cat#: UV-1800; SHIMADU, Japan). The isolated RNA was reverse-transcribed into cDNA using EasyScript One-Step gDNA Removal and cDNA Synthesis SuperMix (Cat#: AE311-03; TransGen Biotech, China). qPCR amplification was performed on a LightCycler®480 II system (Roche, Switzerland) using Hieff qPCR SYBR Green Master Mix (No Rox) (Cat#: 11201ES08; YEASEN, China). The 2^−ΔΔCt^ method was used to determine the RNA expression levels, and the expression levels of circ_0129047/BMPR2 and miR-1206 were normalized using glyceraldehyde-3-phosphate dehydrogenase and uracil 6 as internal controls [51]. All primers used for RT-qPCR are listed in Table 2.

**Table 2.** The primer sequences for RT-qPCR

Name	Primer sequences (5’-3’)
**Circ_0129047**	
Forward	AGGTCCCGTTCTTGTTATCAGT
Reverse	AGCCACTGGAAATTTGAAGCA
**miR-1206**	
Forward	ACGTTGGATGCATGTAGATGTTTAAGCTC
Reverse	CAGTGCAGGGTCCGAGGTAT
**U6**	
Forward	CTCGCTTCGGCAGCACA
Reverse	AACGCTTCACGAATTTGCGT
**BMPR2**	
Forward	GCAGGTTCTCGTGTCTAGGG
Reverse	GTGTGAAGTCCTGCTGTCCA
**ADARB1**	
Forward	TAGAGTCTGGTGAGGGGACG
Reverse	GAGAGGTGGCAGGTCCTCTA
**β-actin**	
Forward	CATGTACGTTGCTATCCAGGC
Reverse	CTCCTTAATGTCACGCACGAT

### Analysis of resistance of circRNAs to RNase R

Total RNA was extracted from A549 and PC9 cells using the TRNzol Universal reagent (Cat#: DP424; TIANGEN, China), as described above, and the total RNA concentration and purity were measured using a SHIMADU UV spectrophotometer (Cat#: UV-1800; SHIMADU, Japan). Then, 4 U/mg RNase R (Cat#: RNR07250, GENESEED, China) was added to 2 g of total RNA, followed by incubation for 30 min at 37°C for linear RNA digestion. After digestion with RNase R, RT-qPCR was performed to analyze the stability of circ_0129047 and linear 0129047 [52].

### Dual-luciferase reporter gene assay

The reporter plasmid vectors, circ_0129047-WT, circ_0129047-Mut, BMPR2 3′-UTR-WT, and BMPR2 3′-UTR-Mut, were purchased from Genecopoeia (China). A549 and PC9 cells (5 × 10^4^ cells/well) were co-transfected with each of these reporter plasmid vectors and miR‐1206 mimic or miR-NC using the Exfect 2000 Transfection Reagent (Cat#: T202-01; Vazyme, China), according to the manufacturer’s instructions. Then, 48 h post-transfection, *Renilla* and firefly luciferase activities were assessed using the Dual Luciferase Reporter Assay Kit (Cat#: DL101-01; Vazyme, China). *Renilla* luciferase was used as an internal reference for firefly luciferase normalization [53].

### RNA immunoprecipitation (RIP) assay

The RIP assay was performed on A549 and PC9 cells using the Magna RIP RNA-Binding Protein Immunoprecipitation Kit (Cat#: 17–700; Sigma-Aldrich, USA) and monoclonal anti-Ago2 antibody (Cat# SAB4200085; Sigma-Aldrich, USA). Briefly, A549 and PC9 cells were transfected with the miR-1206 mimic or miR-NC. At 48 h post transfection, the cells were lysed on ice with RIP lysis buffer containing an RNase inhibitor and protease inhibitor cocktail. The whole supernatant lysate was collected and incubated with RIP buffer containing protein A/G magnetic beads coupled with an anti-IgG antibody or anti-Ago2 antibody at 4°C overnight. Proteinase K was then added to dissolve the protein and isolate the immunoprecipitated RNA. Finally, the co-precipitated RNA was analyzed using RT-qPCR to confirm the presence of binding targets [54].

### Cell viability assay

Cell viability assay was performed to assess the viabilities of A549 and PC9 cells at 0, 24, 48, and 72 h post-transfection using the cell counting kit (CCK)-8 (Cat#: HY-K0301; MedChemExpress, USA). Approximately 5 × 10^3^ A549 and PC9 cells were seeded into each well of a 96-well plate and placed in a 5% CO_2_ incubator at 37°C. After the indicated time points, 10 µL of the CCK-8 reagent was added to each well of the 96-well plate. The plate was then incubated under the same conditions for 2 h, followed by measurement of absorbance at 450 nm on a microplate reader (Cat#: Elx808; Biotek, USA) [55].

### Cell proliferation assay

The bromodeoxyuridine enzyme-linked immunosorbent assay (BrdU-ELISA) was performed to evaluate the proliferation of A549 and PC9 cells using the BrdU Cell Proliferation Kit (Cat#: 2750; Sigma-Aldrich, USA). Approximately 5 × 10^4^ transfected cells were plated into each well of a 96-well plate for 48 h of cultivation. After incubation with BrdU reagent for 4 h, the cells were immobilized by adding a fixing solution to denature the DNA. Next, the anti-BrdU antibody and corresponding secondary antibody were successively incubated for 1 h at room temperature. After reacting with TMB peroxidase substrate, the stop solution was added. The proliferation capacity of cells in each group was determined by measuring the absorbance at 450 nm on a microplate reader (Cat#: Elx808; Biotek, USA) [56].

### Cell apoptosis assay

Caspase-3 colorimetric assay kit (Cat#: ab39401; Abcam, USA) was used for the measurement of caspase-3 activity to evaluate the apoptosis of A549 and PC9 cells 48 h post-transfection. Approximately 2 × 10^5^ transfected A549 and PC9 cells were seeded into each well of a 96-well plate, which was then placed in a 5% CO_2_ incubator at 37°C for 48 h. The cells were lysed with a chilled lysis buffer provided with the kit for 10 min. Then, 50 μL of 2× reaction buffer containing 10 mM dithiothreitol and 5 μL of DEVD-p-NA substrate was added to the supernatant for 2 h at 37°C, followed by measurement of the absorbance at 400 nm on a microplate reader (Cat#: Elx808; Biotek, USA) [57].

### Cell adhesion assay

The adhesion of A549 and PC9 cells was evaluated using a 96-well plate pre-coated with fibronectin (Sigma-Aldrich, USA). Briefly, the plate was coated with 50 µL of fibronectin (20 µg/mL) and incubated overnight at 4°C, followed by blocking with 1% bovine serum albumin for 1 h. Approximately 2 × 10^5^ transfected A549 and PC9 cells were seeded in each well of a 96-well plates and incubated for 1 h at 37°C. The unattached cells were removed, and the attached cells were immobilized with 4% paraformaldehyde, followed by staining with 0.1% crystal violet. Next, 12% sodium dodecyl sulfate was used to dissolve the crystals and the absorbance at 620 nm was determined using a microplate reader (Cat#: Elx808; Biotek, USA) [58].

### Cell migration assay

A wound healing assay was performed to evaluate the migration abilities of A549 and PC9 cells. Briefly, transfected A549 and PC9 cells were inoculated at 5 × 10^4^ cells per well in a 6-well plate and cultivated in an incubator containing 5% CO_2_ at 37°C until a monolayer was formed. The wound was formed by scratching the middle of the cell monolayer with a sterile 20 µL micropipette. This was followed by rinsing with phosphate-buffered saline to remove the cell debris. The cells were then cultured in a serum-free medium under the same conditions for another 24 h. The cells gradually migrated to the wound surface, and the wound areas were photographed at 0 and 24 h using an inverted microscope. The migration ability of the cells in each group was determined by calculating the migration rate using the following formula: (0 h wound width – 24 h wound width)/0 h wound width [59].

### Cell invasion assay

Transwell plates (8 µm; Corning, USA) coated with Matrigel were used to detect the invasion abilities of A549 and PC9 cells. Complete medium containing 20% FBS was added to the lower chamber, and transfected A549 and PC9 cells (5 × 10^4^ cells) were added to the upper chamber. After 24 h, the cells on the lower surface were fixed with methanol for 20 min and stained with 0.5% crystal violet for 15 min. Stained cells were photographed using a microscope (Olympus, Tokyo, Japan) [52].

### RNA pull-down assay

The RNA pull-down assay was performed in A549 and PC9 cells to verify the interaction between BMPR2 mRNA and miR-1206 using a biotin-coupled miR-1206 probe purchased from Sangon Biotech (China). First, the biotin-coupled miR-1206 probe or random oligo probe was incubated with streptavidin magnetic beads (Life Technologies, USA) for 2 h at room temperature, followed by overnight incubation with the lysate from A549 and PC9 cells at 4°C. After that, TRNzol Universal reagent was used to extract the bound RNAs that were pulled down by the biotin-coupled miR-1206 probe, followed by RNA analysis using RT-qPCR.

### Statistical analysis

The experimental results were statistically analyzed using GraphPad Prism 8.0.1 (244) (GraphPad Software, USA). The results of three independent experiments are expressed as the mean ± standard deviation. Significant differences were compared using Student’s *t*-test or analysis of variance. P < 0.05 indicated a significant difference, while P < 0.001 indicated an extremely significant difference.

## Results

In this study, we focused on the effects and action mechanisms of circ_0129047 in LAC. We hypothesized that circ_0129047 inhibited LAC progression by sponging miR-1206 and upregulating BMPR2 expression. Clinical analysis showed that the expression levels of circ_0129047 and BMPR2 were downregulated, while those of miR-1206 were upregulated in LAC. In vitro biological function analysis showed that circ_0129047 or BMPR2 knockdown and miR-1206 overexpression promoted LAC malignant behavior, whereas circ_0129047 or BMPR2 upregulation had the opposite effect. More importantly, we confirmed the relationships among circ_0129047, miR-1206, and BMPR2 in LAC.

### Identification of the circ_0129047/miR-1206/BMPR2 axis in LAC

Two mRNA expression profiles (GSE118370 and GSE85841) from the Gene Expression Omnibus (GEO) Datasets were used to select the differentially expressed genes (DEGs) with adj.P value < 0.05 (Figure 1a). After uploading the 364 common DEGs from GSE118370 and GSE85841 to the Search Tool for the Retrieval of Interacting Genes/Proteins (STRING) and Metascape for gene ontology (GO) enrichment, we found that 50 DEGs were associated with the regulation of cell migration, while 34 DEGs were associated with the negative regulation of cell proliferation (Figure 1b, c). Eleven key genes were selected by overlapping the results of STRING and Metascape (Figure 1d). Based on the analysis using The Cancer Genome Atlas database, the expression levels of activin A receptor-like type 1, adenosine deaminase RNA-specific B1 (*ADARB1), BMPR2*, and DLC1 Rho GTPase activating protein were found to be significantly downregulated in LAC (Figure 1e). Among these four genes, low expression of *ADARB1* and *BMPR2* was associated with poor prognosis according to the Kaplan–Meier analysis (figure 1f). In GEPIA database, both ADARB1 and BMPR2 were downregulated in tumor samples (Figure 1g). We then found that the mRNA expression levels of *BMPR2* were lower than those of *ADARB1* in the tissues of 37 patients with LAC; hence, *BMPR2* was identified as the gene of interest (Figure 1h). After downloading the circRNA expression profile (GSE112214) from GEO Datasets, circ_0129047, which showed the lowest expression in LAC samples, was screened out (Figure 1i). The structure of circ_0129047 is shown in Figure 1j. The miRNAs binding to BMPR2 and circ_0129047 were predicted using TargetScan and Circular RNA Interactome, respectively, and the upregulated miRNAs were screened from the miRNA expression profile, GSE68951, with adj. P value < 0.05, and log_2_FC > 0. Finally, only miR-1206 was found to overlap between the two sets of results obtained (Figure 1k).

**Figure 1.** **The identification of circ_0129047/miR-1206/BMPR2 axis in LAC**. (a) 364 DEGs were overlapped from GSE118370 and GSE85841 with adj.P value <0.05. GSE118370 and GSE85841 were two mRNA expression profiles. (b) The GO enrichment of 364 DEGs was analyzed by STRING. (c) The GO enrichment of 364 DEGs was analyzed by Metascape. (d) 11 key genes involving cell migration and cell proliferation were selected. (e) The expression levels of 11 genes in LAC were analyzed by TCGA database. (f) The prognosis of four downregulated genes was analyzed by Kaplan-Meier Plotter. (g) GEPIA database displayed the expression of ADARB1 and BMPR2 in tumor and normal samples. LUAD, lung adenocarcinoma. *P < 0.01. (h) The levels of ADARB1 and BMPR2 in our collected clinical samples were detected by RT-qPCR. (i) The top 5 downregulated circRNAs in LAC were screened from GSE112214. GSE112214, circRNAs expression profile. (j) The structure of circ_0129047. (k) miR-1206 with high expression in LAC were selected from GSE68951, as well as it could binding to BMPR2 and circ_0129047.

### Characterization of circ_0129047 in LAC

To explore the role of circ_0129047, we characterized the main trend of circ_0129047 expression in LAC. First, 37 paired LAC and adjacent normal tissue samples were used to determine the expression levels of circ_0129047 using RT-qPCR. As shown in Figure 2a, the expression levels of circ_0129047 decreased by 50% on an average in LAC tissues when compared with those in adjacent normal tissues. In addition, the expression levels of circ_0129047 were measured via RT-qPCR in five LAC cell lines (A549, Calu-3, H1975, PC9, and SPC-A1) and one non-cancer cell line (BEAS-2B). Similar to the results for tissue analysis, the expression levels of circ_0129047 in five LAC cell lines were lower than those in the non-cancer cell line, and the expression of circ_0129047 was the most downregulated in A549 and PC9 cell lines (Figure 2b). Hence, A549 and PC9 cell lines were selected for subsequent functional experiments. A549 and PC9 cell lysates were treated with RNase R to assess the stability of circ_0129047 and linear 0129047. The results showed that after RNase R treatment, the levels of linear 0129047 decreased by approximately 80%, while those of circ_0129047 did not change, indicating that circ_0129047 had an anti-digestion effect against RNase R (Figure 2c). To assess the subcellular localization of circ_0129047 and linear 0129047 in A549 and PC9 cells, the expression levels of these two types of RNAs were measured in the nucleus and cytoplasm. We found that both circ_0129047 and linear 0129047 were principally distributed in the cytoplasm of A549 and PC9 cells (Figure 2d). Together, these data demonstrate that circ_0129047 principally exists in the cytoplasm as a circular and stable transcript, and shows reduced expression in LAC.

**Figure 2.** **Characterization of circ_0129047 in LAC**. (a) RT-qPCR analysis was carried out for circ_0129047 expression in human LAC tissues and adjacent normal tissues, n = 37, Student’s *t*-test. (b) RT-qPCR analysis was carried out for circ_0129047 expression in different of human LAC cell lines (A549, Calu-3, H1975, H460, and PC9) and normal human bronchial epithelial cell line (Beas-2B), *P < 0.05, **P < 0.001 compared with Beas-2B cell line, ANOVA. (c) The expression of circ_0129047 and linear 0129047 were detected by RT-qPCR in A549 and PC9 cells with or without RNase R treatment, **P < 0.001, ANOVA. (d) The nuclear and cytoplasmic RT-qPCR was carried out to verify subcellular localization of circ_0129047 and linear 0129047 in A549 and PC9 cells, **P < 0.001, Student’s *t*-test. Data were from three independent experiments and presented as the mean ± SD.

### Circ_0129047 silencing facilitates the malignant phenotype of LAC cells

Next, we verified the role of circ_0129047 in the biological functions of LAC cells. A549 and PC9 cells were transfected with circ_0129047 siRNA, and the results showed that circ_0129047 levels in the si-circ group were reduced by more than 70% compared to those in the si-NC group (Figure 3a). Subsequently, the functions of circ_0129047 in A549 and PC9 cells were analyzed by evaluating the cell viability, proliferation, apoptosis, adhesion, migration, and invasion. CCK-8 assay showed that the viability of A549 and PC9 cells increased by more than 1.3 times after the downregulation of circ_0129047 expression (Figure 3b). BrdU-ELISA showed that circ_0129047 silencing upregulated the proliferation of A549 and PC9 cells by 1.4-fold (Figure 3c). In addition, to evaluate the effect of circ_0129047 on apoptosis, caspase-3 activity was measured in LAC cells, and the results showed that the downregulation of circ_0129047 expression reduced caspase-3 activity by nearly 55% (Figure 3d). Cell adhesion in the si-circ group increased by approximately 1.5 times compared to that in the si-NC group (Figure 3e). The wound healing and Transwell experiments showed that the migration and invasion abilities of LAC cells in the si-circ group were 2 and 2.2 times higher than those in the si-NC group, respectively (figure 3f and 3g). Functional experiments revealed that low circ_0129047 expression promoted the viability, proliferation, adhesion, migration, and invasion, while inhibiting the apoptosis of LAC cells.

**Figure 3.** **Circ_0129047 silencing facilitated malignant phenotypes of LAC cells**. (a) RT-qPCR analysis was carried out for circ_0129047 expression in A549 and PC9 cells transfected with circ_0129047 siRNA. (b) CCK-8 assay was carried out for detection the viability of A549 and PC9 cells transfected with circ_0129047 siRNA. (c) BrdU proliferation assay was carried out for detection the proliferation of A549 and PC9 cells transfected with circ_0129047 siRNA. (d) Caspase-3 activity assay was carried out for detection the apoptosis of A549 and PC9 cells transfected with circ_0129047 siRNA. (e) Cell adhesion assay was carried out for assessment the adhesion ability of A549 and PC9 cells transfected with circ_0129047 siRNA. (f) Wound healing assay was carried out for assessment the migration ability of A549 and PC9 cells transfected with circ_0129047 siRNA. (g) Transwell assay was carried out for assessment the invasion ability of A549 and PC9 cells transfected with circ_0129047 siRNA. Si-circ: circ_0129047 siRNA, *P < 0.05, **P < 0.001 compared with control group, ANOVA. Data were from three independent experiments and presented as the mean ± SD.

### Circ_0129047 serves as a sponge of miR-1206 in LAC cells

CircRNAs act as sponges for miRNAs to exert their unique regulatory roles [60]. We hypothesized that miR-1206 could be a target for circ_0129047, and the predicted binding sites between them are shown in Figure 4a. We confirmed this hypothesis using dual-luciferase reporter assays. As shown in Figure 4b, compared with miR-NC, co-transfection of the miR-1206 mimic in A549 and PC9 cells resulted in a 60% decrease in luciferase activity of the wild-type circ_0129047 reporter vector, while there was no prominent difference in the luciferase activity of the mutant circ_0129047 reporter vector, suggesting an interplay between circ_0129047 and miR-1206. A549 and PC9 cells were subjected to the Ago2-RIP assay to further confirm the interplay between circ_0129047 and miR-1206. As illustrated in Figure 4c, when the miR-1206 mimic was transfected into A549 or PC9 cells, circ_0129047 levels were elevated in the anti-Ago2 group than in the anti-IgG group, suggesting that miR-1206 and circ_0129047 existed in the same RNA-induced silencing complex. Additionally, the expression levels of miR-1206 were elevated in LAC tissues, being four times higher than those in the adjacent normal tissues (Figure 4d). According to the Pearson correlation analysis, an inverse association between miR-1206 and circ_0129047 expression levels were observed in LAC tissues (Figure 4e). Overall, these findings suggest that circ_0129047 acts as a sponge for miR-1206 and negatively modulates miR-1206 expression in LAC.

**Figure 4.** **Circ_0129047 served as a sponge of miR-1206 in LAC cells**. (a) Schematic diagram of circ_0129047 with miR-1206 binding sites predicted by TargetScan. (b) Dual-luciferase reporter assay was carried out to verify the relationship between circ_0129047 and miR-1206 in A549 and PC9 cells co-transfected with wild-type or mutant circ_0129047 luciferase reporter vector and miR-1206 mimic or miR-NC, circ-WT: wild-type circ_0129047, circ-Mut: mutant circ_0129047, **P < 0.001, ANOVA. (c) RIP assay was carried out using anti-Ago2 antibody or anti-IgG antibody in A549 and PC9 cells transfected with miR-1206 mimic or miR-NC, followed by RT-qPCR analysis for circ_0129047 expression, **P < 0.001 compared with the miR-NC and IgG group, ANOVA. (d) RT-qPCR analysis was carried out for miR-1206 expression in human LAC tissues and adjacent normal tissues, n = 37, Student’s *t*-test. (e) Correlation between circ_0129047 and miR-1206 expression in 37 human LAC tissues was determined by Pearson correlation analysis.

### Circ_0129047 overexpression suppresses the malignant phenotype of LAC cells by inhibiting the expression of miR-1206

We evaluated the potential functions of miR-1206 and circ_0129047 in LAC by transfecting the circ_0129047 overexpression vector, miR-1206 mimic, or both into A549 and PC9 cells. Transfection efficiency was verified using RT-qPCR prior to functional experiments. As shown in Figure 5a, the expression levels of circ_0129047 were increased by 2-fold after transfection with the circ_0129047 overexpression vector, while the miR-1206 mimic caused the expression levels of miR-1206 to increase by 2.5-fold. The overexpression of circ_0129047 could lead to the downregulation of miR-1206 expression, but the upregulation of miR-1206 expression had no significant effect on the expression of circ_0129047. CCK-8 assay revealed that the viabilities of A549 and PC9 cells were reduced by the upregulation of circ_0129047 expression and promoted by the upregulation of miR-1206 expression. Notably, the miR-1206 mimic partly alleviated the inhibitory effect of circ_0129047 overexpression on the viabilities of A549 and PC9 cells when co-transfected with the circ_0129047 overexpression vector (Figure 5b). The proliferation of A549 and PC9 cells was monitored using BrdU ELISA, and the results revealed that A549 and PC9 cells showed a 40% decrease in cell proliferation after circ_0129047 overexpression and a 50% increase in cell proliferation after miR-1206 overexpression. The suppression of cell proliferation mediated by circ_0129047 overexpression could be partly restored by miR-1206 overexpression (Figure 5c). In addition, to evaluate the effects of miR-1206 and circ_0129047 on cell apoptosis, we examined the caspase-3 activity in A549 and PC9 cells and found that circ_0129047 overexpression enhanced the caspase-3 activity by nearly 5 times, whereas miR-1206 overexpression decreased the caspase-3 activity by approximately 60%. After co-transfection, there were no distinct changes in caspase-3 activity, suggesting that circ_0129047 plays a role in accelerating apoptosis, while miR-1206 plays a role in impeding apoptosis (Figure 5d). In addition, cell adhesion assay revealed that circ_0129047 overexpression reduced the adhesion of A549 and PC9 cells by approximately 40%, while miR-1206 overexpression increased the adhesion of A549 and PC9 cells by approximately 65%, while no changes were observed in the adhesion of A549 and PC9 cells in the co-transfection group (Figure 5e). Furthermore, the wound healing assay revealed that circ_0129047 overexpression led to an approximately 60% decrease, while miR-1206 overexpression led to an approximately 30% increase in the migration abilities of A549 and PC9 cells, and no obvious changes were observed in the co-transfection group (figure 5f). Similarly, transwell analysis showed that the invasion of circ_0129047-overexpressing A549 and PC9 cells was reduced by approximately 40%, while that of miR-1206-overexpressing cells was increased by approximately 2.5 times, reversing the invasion-inhibiting effect of circ_0129047 overexpression (Figure 5g). In summary, functional experiments revealed that circ_0129047 inhibits, while miR-1206 promotes the malignant phenotype of LAC cells.

**Figure 5.** **Circ_0129047 overexpression suppressed malignant phenotypes of LAC cells by inhibiting the expression of miR-1206**. (a) RT-qPCR analysis was carried out for circ_0129047 and miR-1206 expression in A549 and PC9 cells transfected with circ_0129047-OE vector, miR-1206 mimic or both. (b) CCK-8 assay was carried out for detection the viability of A549 and PC9 cells transfected with circ_0129047-OE vector, miR-1206 mimic or both. (c) BrdU proliferation assay was carried out for detection the proliferation of A549 and PC9 cells transfected with circ_0129047-OE vector, miR-1206 mimic or both. (d) Caspase-3 activity assay was carried out for detection the apoptosis of A549 and PC9 cells transfected with circ_0129047-OE vector, miR-1206 mimic or both. (e) Cell adhesion assay was carried out for assessment the adhesion ability of A549 and PC9 cells transfected with circ_0129047-OE vector, miR-1206 mimic or both. (f) Wound healing assay was carried out for assessment the migration ability of A549 and PC9 cells transfected with circ_0129047-OE vector, miR-1206 mimic or both. (g) Transwell assay was carried out for assessment the invasion ability of A549 and PC9 cells transfected with circ_0129047-OE vector, miR-1206 mimic or both. circ-OE: circ_0129047 overexpression, mimic: miR-1206 mimic, *P < 0.05, **P < 0.001 compared with control group, ^#^P < 0.05, ^##^P < 0.001 compared with the circ_0129047-OE + miR-1206 mimic group, ANOVA. Data were from three independent experiments and presented as the mean ± SD.

### BMPR2 *is a downstream target gene of miR-1206 in LAC*

miRNAs function by binding to the 3′-UTRs of their target mRNAs [61]. Thus, we attempted to identify the downstream targets of miR-1206 using miRanda (http://www.microrna.org/). We focused on BMPR2 whose 3′-UTR contains a potential binding site for miR-1206, as displayed in Figure 6a. To validate our prediction, we performed a dual-luciferase reporter assay in A549 and PC9 cells and revealed that enforced expression of miR-1206 resulted in an approximately 65% reduction in luciferase activity of the reporter vector containing the wild-type BMPR2 3′-UTR sequence, while it had no effect on the luciferase activity of the mutant reporter vector (Figure 6b). In addition, RNA pull-down assays were performed on A549 and PC9 cells. As illustrated in Figure 6c, an approximately 6-fold enrichment of BMPR2 mRNA by biotin-coupled miR-1206 probe was detected in A549 and PC9 cells compared with the enrichment by NC probe, suggesting that miR-1206 could directly bind to BMPR2 mRNA. Furthermore, we observed a clear inverse association between miR-1206 and BMPR2 mRNA expression levels in LAC tissues (Figure 6d). Taken together, the data in this section revealed that BMPR2 acts as a downstream target gene of miR-1206 and directly binds to it in LAC.

**Figure 6.** **BMPR2 was the downstream target of miR-1206 in LAC**. (a) Schematic diagram of the predicted miR-1206 binding sites in the 3’-UTR of BMPR2 mRNA. (b) Dual-luciferase reporter assay was carried out to verify the relationship between BMPR2 mRNA and miR-1206 in A549 and PC9 cells co-transfected with wild-type or mutant BMPR2 mRNA 3’-UTR luciferase reporter vector and miR-1206 mimic or miR-NC, WT: wild-type BMPR2 mRNA 3’-UTR, Mut: mutant BMPR2 mRNA 3’-UTR, **P < 0.001, ANOVA. (c) RNA pull-down assay was carried out using biotin-coupled miR-1206 probe or oligo probe in the A549 and PC9 cells, followed by RT-qPCR analysis for BMPR2 mRNA expression, **P < 0.001, Student’s *t*-test. (d) Correlation between miR-1206 and BMPR2 mRNA expression in 37 human LAC tissues was determined by Pearson correlation analysis.

### BMPR2 knockdown aggravates the malignant phenotype of LAC cells

Next, we investigated the effect of low expression of BMPR2 on LAC cells. RT-qPCR showed that the BMPR2 levels in the si-BMPR2 group decreased by approximately 80% compared to those in the si-NC group in LAC cells (Figure 7a). CCK-8 and BrdU assays showed that BMPR2 knockdown increased the viability and proliferation of LAC cells by approximately 1.3 times and 1.5 times, respectively (Figure 7b and 7c). In addition, caspase-3 activity analysis revealed approximately 50% downregulation of caspase-3 activity in BMPR2 knockdown cells (Figure 7d). As expected, adhesion, migration, and invasion of A549 and PC9 cells were enhanced in the si-BMPR2 group compared with their values in the si-NC group (Figure 7e, 7f, and 7g). In summary, these results suggest that BMPR2 knockdown promotes the malignant behavior of LAC cells.

**Figure 7.** **BMPR2 knockdown aggravated the malignant phenotypes of LAC cells**. (a) RT-qPCR analysis was carried out for BMPR2 mRNA expression in A549 and PC9 cells transfected with BMPR2 siRNA. (b) CCK-8 assay was carried out for detection the viability of A549 and PC9 cells transfected with BMPR2 siRNA. (c) BrdU proliferation assay was carried out for detection the proliferation of A549 and PC9 cells transfected with BMPR2 siRNA. (d) Caspase-3 activity assay was carried out for detection the apoptosis of A549 and PC9 cells transfected with BMPR2 siRNA. (e) Cell adhesion assay was carried out for assessment the adhesion ability of A549 and PC9 cells transfected with BMPR2 siRNA. (f) Wound healing assay was carried out for assessment the migration ability of A549 and PC9 cells transfected with BMPR2 siRNA. (g) Transwell assay was carried out for assessment the invasion ability of A549 and PC9 cells transfected with BMPR2 siRNA. Si-BMPR2: BMPR2 siRNA, *P < 0.05, **P < 0.001 compared with control group, ANOVA. Data were from three independent experiments and presented as the mean ± SD.

### miR-1206 overexpression contributes to the malignant phenotype of LAC cells by inhibiting the expression of BMPR2

Given the interaction between miR-1206 and BMPR2, we hypothesized that the promoting effect of miR-1206 on LAC progression was achieved by inhibiting BMPR2 expression. Therefore, we explored the effects of BMPR2 on the malignant cell phenotypes of A549 and PC9 cells by transfecting them with the BMPR2 overexpression vector, miR-1206 mimic, or both. The transfection of BMPR2 overexpression vector successfully increased the expression levels of BMPR2 by approximately 3.2 times (Figure 8a). Transfection with the miR-1206 mimic decreased BMPR2 expression levels by 40%. However, co-transfection with the BMPR2 overexpression vector and miR-1206 mimic did not have any significant effect on BMPR2 expression levels. CCK-8 assay showed that the viabilities of A549 and PC9 cells were weakened by BMPR2 overexpression, and this effect was recovered by the miR-1206 mimic (Figure 8b). Likewise, the proliferation of A549 and PC9 cells was restrained by BMPR2 overexpression, which was reversed by the miR-1206 mimic, as determined by BrdU-ELISA (Figure 8c). Besides, BMPR2 overexpression increased the caspase-3 activity of A549 and PC9 cells by approximately 5 times, which was abrogated by the miR-1206 mimic (Figure 8d). In addition, BMPR2 overexpression reduced the adhesion of A549 and PC9 cells by approximately 40%, which was partially rescued by the miR-1206 mimic (Figure 8e). Furthermore, the migration capacity of A549 and PC9 cells changed in a consistent manner, as determined by the wound healing assay. As illustrated in figure 8f, the migration capacities of A549 and PC9 cells in the BMPR2-OE group were reduced by 56%, whereas the BMPR2-OE + miR-1206 mimic group showed no obvious change. Transwell analysis revealed more than 50% reduction in cell invasion in the BMPR2-overexpressing group, and this effect was partially eliminated by the miR-1206 mimic (Figure 8g). Together, these findings indicate that the functions of miR-1206 and BMPR2 in LAC progression are antagonistic, and that miR-1206 overexpression contributes to the malignant phenotype of LAC cells by inhibiting BMPR2 expression.

**Figure 8.** **MiR-1206 overexpression contributed to the malignant phenotypes of LAC cells by inhibiting the expression of BMPR2**. (a) RT-qPCR analysis was carried out for miR-1206 and BMPR2 mRNA expression in A549 and PC9 cells transfected with BMPR2-OE vector, miR-1206 mimic or both. (b) CCK-8 assay was carried out for detection the viability of A549 and PC9 cells transfected with BMPR2-OE vector, miR-1206 mimic or both. (c) BrdU proliferation assay was carried out for detection the proliferation of A549 and PC9 cells transfected with BMPR2-OE vector, miR-1206 mimic or both. (d) Caspase-3 activity assay was carried out for assessment the apoptosis of A549 and PC9 cells transfected with BMPR2-OE vector, miR-1206 mimic or both. (e) Cell adhesion assay was carried out for assessment the adhesion ability of A549 and PC9 cells transfected with BMPR2-OE vector, miR-1206 mimic or both. (f) Wound healing assay was carried out for assessment the migration ability of A549 and PC9 cells transfected with BMPR2-OE vector, miR-1206 mimic or both. (g) Transwell assay was carried out for assessment the invasion ability of A549 and PC9 cells transfected with BMPR2-OE vector, miR-1206 mimic or both. BMPR2-OE: BMPR2 overexpression, mimic: miR-1206 mimic, *P < 0.05, **P < 0.001 compared with control group, ^#^P < 0.05, ^##^P < 0.001 compared with the BMPR2-OE + miR-1206 mimic group, ANOVA. Data were from three independent experiments and presented as the mean ± SD.

## Discussion

In our study, we identified the inhibitory effect of circ_0129047 on LAC for the first time. We compared LAC tissues with adjacent normal tissues and found that in tumor tissues, the expression levels of circ_0129047 and BMPR2 were decreased, while those of miR‐1206 were elevated. Subsequent experiments showed that the overexpression of circ_0129047 and BMPR2 accelerated LAC cell apoptosis and prominently suppressed the viability, proliferation, adhesion, migration, and invasion of LAC cells. These effects were reversed by the knockdown of miR-1206 mimic, circ_0129047, or BMPR2. In summary, this study revealed that circ_0129047 acts as a sponge of miR-1206 to upregulate BMPR2 expression by downregulating miR-1206 expression, thereby inhibiting LAC progression.

CircRNAs play important roles in oncogenesis and tumor cell malignant behavior as activators or suppressors of LAC. For example, hsa_circ_002503 acts as a tumor-promoting circRNA whose expression is upregulated in LAC, and its knockdown inhibits the proliferation and promotes the apoptosis of LAC cells [62]. The expression levels of hsa_circ_0002346 are low in LAC samples, and it can inhibit the invasion and metastasis of LAC cells *in vitro* and *in vivo* [63]. Yao *et al*. [17] reported the downregulation of circ_0006427 expression in LAC tissues and proved that circ_0006427 inhibited cell proliferation, migration, invasion, and epithelial–mesenchymal transformation progression *in vitro*, while also inhibiting tumor growth and metastasis *in vivo*. However, many circRNAs still need to be identified, and their roles in LAC need to be further studied. In this study, we identified a novel circRNA, circ_0129047, with low expression levels in LAC cells and tissues. Our data revealed that circ_0129047 significantly induced LAC cell apoptosis *in vitro*, and had clear inhibiting effects on the viability, proliferation, adhesion, and migration of LAC cells.

Our findings suggest that circ_0129047, as a tumor suppressor, may play unexpected roles in the carcinogenesis and development of LAC. Our results for circ_0129047 appear to be consistent with those for circ_0006427 and hsa_circ_0002346 in LAC.

CircRNAs act as sponges for miRNAs to exert their unique regulatory roles [64]. CircRNAs localized to different parts of the cell perform different functions, and circRNA cytoplasmic localization is closely related to the sponging effect on miRNA [12,65]. We hypothesized that cytoplasmic localized circ_0129047 may play a role in LAC. Our experiments confirmed this hypothesis and revealed miR-1206 as the target of circ_0129047. Additionally, miR-1206 overexpression significantly promoted the malignant phenotype of LAC cells. In summary, miR-1206, as a tumor promoter, participates in the oncogenesis and development of LAC. Our findings are similar to those of previous studies on the expression of miR-1206 in Burkitt’s lymphoma. Konrad Huppi *et al*. [30] found that miR-1206 was highly expressed in Burkitt lymphoma cells (Namalwa and CA46) than in normal peripheral blood lymphocytes. Interestingly, some members of the 8q24 miRNA cluster, miR-1205, miR-1207-3p, miR-1207-5p, and miR-1208, were highly expressed in approximately 50% of gastric cancer tissues compared to their expression in adjacent non-tumor tissues, while no or little expression of miR-1206 was detected in the cancerous and non-cancerous gastric tissues as well as gastric cancer cell lines [31]. This suggests that miR-1206 may play different roles in different cancer types.

miRNAs regulate gene expression by binding to the 3′-UTRs of downstream target mRNAs [66]. Through their interaction with mRNAs, miRNAs inhibit mRNA translation and/or cleavage, eventually leading to the downregulation of protein expression [67]. In our study, we demonstrated that miR-1206 directly targeted BMPR2. Moreover, our study revealed that BMPR2 was weakly expressed in LAC tissues and overexpression of BMPR2 inhibited the viability, proliferation, adhesion, and migration of LAC cells, while inducing LAC cell apoptosis. Furthermore, BMPR2 silencing facilitated the malignant behavior of LAC cells. Our findings are consistent with those of previous studies. BMPR2 acts as a tumor suppressor in some cancer types. Overexpression of BMPR2 inhibits, while short hairpin RNA-mediated knockdown of BMPR2 promotes the cell proliferation and clonal formation of neuroblastoma cells [48]. Tao *et al*. [68] revealed that BMPR2 interference suppresses the proliferation of osteosarcoma cells, while promoting their apoptosis and cellular radiosensitivity. Kettunen *et al*. [50] demonstrated the downregulation of BMPR2 expression levels in 13 squamous cell lung cancer tissues and 13 LAC tissues compared to those in the normal lung tissues.

## Conclusions

The present study is the first to report circ_0129047 as a cancer-suppressing circRNA whose expression levels are decreased in LAC tissues and cells, and it inhibits the viability, proliferation, adhesion, migration, and invasion, while inducing the apoptosis of LAC cells. Our study also found that BMPR2 expression levels were downregulated, while those of miR-1206 were upregulated in LAC tissues. Circ_0129047 acted as a sponge of miR-1206 and upregulated BMPR2 expression to inhibit the malignant phenotype of LAC cells. These results suggest a new mechanism for the progression of LAC that should be investigated further in future studies.

## Supplementary Material

Supplemental Material

## Data Availability

The datasets used and/or analyzed during the current study are available from the corresponding author on reasonable request.
